The article "Effect of Noni on Memory Impairment Induced by Hydrocortisone in Mice" was published in 2022. Journal: Evid Based Complement Alternat Med.

# Effect of Noni on Memory Impairment Induced by Hydrocortisone in Mice

**DOI:** 10.1155/2022/2781906

**Published:** 2022-09-08

**Authors:** Rui Zhang, Jinlian Liu, Songrui Di, Shuhui Yu, Xinjuan Hou, Fan Zhao, Chandi Wang, Yingli Zhu, Ruying Tang, Shixin Deng, Chun Wang, Jianjun Zhang

**Affiliations:** ^1^School of Traditional Chinese Medicine, Beijing University of Chinese Medicine, Beijing 100029, China; ^2^School of Chinese Materia Medica, Beijing University of Chinese Medicine, Beijing 100029, China; ^3^Department of Research and Development, NewAge Incorporated, American Fork, UT 84003, USA

## Abstract

**Background:**

Oxidative stress and memory impairment have been implicated as common functional brain diseases. Nuclear factor E2-related factor 2 (Nrf2) is highly induced in oxidative stress, indicating that Nrf2 is an emerging target of memory therapy. This study aimed to investigate the effect of noni on brain memory impairment induced by hydrocortisone and its protective mechanism in mice.

**Methods:**

Male Kunming mice (*n* = 8/group) were given hydrocortisone by gastric gavage for 14 consecutive days to establish the memory impairment model, except for those in the control group. On the same day, the corresponding drugs were given by gastric gavage. The changes in ethology were examined. The brains were extracted and subjected to western blot analysis and biochemical analyses to assess the activities of antioxidative stress.

**Results:**

The middle- and high-dose noni groups exhibited ameliorated ethology, and the high-dose noni group exhibited increased cerebral protein expression of Nrf2, Kelch-like ECH-associated protein 1 (KEAP1), and haem oxygenase-1 (HO-1) compared to the model group. The arrangement of CA3 vertebral cells in the hippocampus of mice was slightly compact, and hyperchromasia and pyknosis were alleviated. Furthermore, biochemical analyses showed that the activities of enzymes related to oxidative stress in the high-dose noni group were increased.

**Conclusions:**

Noni might be a powerful antioxidant that can protect nerve cells and may possess potential benefits for the treatment of memory impairment.

## 1. Introduction

*Morinda citrifolia* Linn (noni) is widely distributed in the southern Pacific Islands and the Indo-China Peninsula, where it has been used traditionally in several herbal remedies for the management of various kinds of diseases, such as wounds, infections, pain, diarrhoea, and mosquito bites [1, 2]. In 2010, noni puree was approved as a new resource food by the Ministry of Health of China for the first time. Since being introduced, noni has been cultivated in the Hainan and Yunnan provinces of China. Moreover, some related beverages, such as Xisha Noni® and Mornida®, have been widely used, and several dietary supplements that contain traditional Chinese functional foods, such as *Panax ginseng*, *Ligustrum lucidum* Ait, *and Cornus officinalis* Sieb, have been employed. According to our methodology and a previous study, noni's traditional Chinese medicine property was summarized and given [3, 4]. Noni, as a new foreign remedy introduced to traditional Chinese medicine, has gradually received more attention.

The article "Effect of Noni on Memory Impairment Induced by Hydrocortisone in Mice" was published in 2022. Journal: Evid Based Complement Alternat Med.

Recent studies suggest that noni has beneficial effects in improving memory functions in mice by reducing oxidative stress and increasing brain levels of brain-derived neurotrophic factor, acetylcholine, and ATP [5, 6]. Noni extract inhibited activity against acetylcholine esterase and monoamine oxidase, and the consequent increase in dopamine and serotonin levels in mice [7]. Noni can ameliorate cerebral blood flow, oxidative stress, and acetylcholinesterase activity in scopolamine-induced memory-impaired mice [8]. It shows a strong antioxidant capacity in the clinic by reducing the superoxide anion radicals, lipid hydroperoxide levels, and lipid peroxidation-derived DNA adduct levels, which were attributable to the antioxidant properties [9, 10]. However, the complete mechanism is still not known. Oxidative stress is a major factor involved in the development and progression of dementia, which is closely related to oxidative stress [11, 12]. Excessive oxidative stress is known to inflict neuronal damage leading to impaired brain functions [13]. It has been reported that oxidative stress is related to the Nrf2/KEAP1/HO-1 pathway [14]. Nuclear factor E2-related factor 2 (Nrf2) is an essential regulator that induces the gene expression of phase II enzymes, and haem oxygenase-1 (HO-1) among the phase II enzymes has a protective effect on cells [15]. In our study, the powerful antioxidant capacity of noni was the breakthrough point leading to the exploration of its mechanism, which could improve memory and provide an experimental basis for the further development of memory products.

In this study, we investigated the effect of noni on memory impairment induced by hydrocortisone in mice to investigate the mechanism of the neuroprotective effect, with particular emphasis on brain oxidative stress.

## 2. Methods

### 2.1. Experimental Animals

Forty-eight healthy male Kunming mice, weighing 20 ± 2 g, were provided by SPF (Beijing) Biotechnology Company Limited (animal qualification certificate No. SCXK (Jing)-2016-0002) and were allowed to acclimatize for 3 days before the experiment. The mice were housed 4 per cage and maintained under a 12 : 12-h light/dark cycle at 55% humidity and 22 ± 2°C with free access to food and water. Procedures involving mice were approved by the Institutional Animal Care and Use Committee of the Beijing University of Chinese Medicine (BUCM-4-2019010201-1096). All procedures were performed in strict accordance with the recommendations in the Guide for the Care and Use of Laboratory Animals of the National Institutes of Health. The study was carried out in compliance with the ARRIVE guidelines.

The article "Effect of Noni on Memory Impairment Induced by Hydrocortisone in Mice" was published in 2022. Journal: Evid Based Complement Alternat Med.

### 2.2. Drugs, Reagents, and Instruments

The dry powder of noni puree was provided by Morinda Inc. The Noni powder was suspended in water and prepared to a concentration of 0.5 mg/10 mL. Hydrocortisone injection was provided by TianJin KingYork Ltd. (CAT H12020887). Acetylcholine (ACh), 5-Hydroxytryptamine (5-HT), dopamine (DA), and noradrenaline (NA) ELISA kits were purchased from Jiangsu Meimian Industrial Co., Ltd. (CAT MB3256B, MB3179B, MB3092B, and MB3269B). Total superoxide dismutase (T-SOD), catalase (CAT), lipid peroxidation (LPO), and malondialdehyde (MDA) kits were purchased from the Nanjing Jiancheng Bioengineering Institute (CAT A001-1-1, A007-1-1, A106-1-2, and A003-1-1). Anti-Nrf2, anti-KEAP1, anti-HO-1, and anti-*β*-actin were purchased from Bioss (Beijing, China) (CAT BJ07138310, BJ07012178, BJ02265489, and AH11286487).

### 2.3. Grouping, Modelling, and Experimental Design

Forty-eight male Kunming mice were divided into 6 groups using a random number table, with 8 in each group: the control group, the model group (double distilled water 10 mL/kg/day), the ginseng group (1 g/kg/day), the high-dose noni group (1.33 g/kg/day, H-noni), the middle-dose noni group (0.67 g/kg/day, M-noni), and the low-dose noni group (0.33 g/kg/day, L-noni). In the morning, forty rats were given hydrocortisone (25 mg/kg/day) by gastric gavage for 14 consecutive days to establish the memory impairment model [16], except for those in the control group. On the same day, the corresponding drugs were administered by gastric gavage in the afternoon. The weight, brain index, and behaviour of the mice in each group were observed. There were no accidental deaths among the mice during the experiment. After the experiment, the mice were killed by cervical dislocation, and left brain tissues were separated and stored at –80°C for analysis.

### 2.4. Measurement of the Mouse Body Weight and the Brain Index

Each mouse was weighed weekly. The wet weight of the brain tissue was measured using a balance, and the brain index (BI) was calculated as follows: BI = brain wet weight/mouse weight × 100%.

### 2.5. Ethics Assessments

The ethology was assessed with the step-down test and passive avoidance test. The incubation period was defined as the time from when the mice were placed on the insulated platform in the box to the first time they jumped off the platform. The training phase occurred after 3 min of acclimatization in a dark box, the mice were stimulated with an immediate 36 V alternating current, and then placed on the platform for an acclimatization period. The incubation period and the number of errors in jumping off the platform within 5 min were recorded. After 5 d of cessation of training, the vanish test was performed. The incubation period was the time from the time each mouse was placed in the open chamber to the time when it was first shocked in the dark chamber. Since mice are nocturnal animals and instinctively flee to the dark, electric shock was used to train their spatial learning and memory. In the training phase, each mouse was put into the open chamber, the door was raised after 5 s, the door was closed as soon as the animal entered the dark chamber completely, and an unavoidable electric shock of 36 V was delivered to the mouse's feet for 2 s. Then, the mouse was moved to the open chamber, and the process was repeated after 5 min. The training was terminated when the mice remained in the light room for 5 min. Twenty-four hours later, the incubation period and the number of errors in entering the dark room within 5 min were recorded for each mouse. The training was stopped for 5 d, and the vanish test was performed.

The article "Effect of Noni on Memory Impairment Induced by Hydrocortisone in Mice" was published in 2022. Journal: Evid Based Complement Alternat Med.

### 2.6. Brain Histology

The right brain tissues were fixed in 4% paraformaldehyde buffer for 36 h and embedded in paraffin. Sections were cut at 4.0 *μ*m and stained with haematoxylin and eosin (HE staining) for histopathologic examinations using standard protocols. All of the images were acquired using a digital pathology system Axio Scan. Z1 (Zeiss, Germany) for assessing the nerve cells.

### 2.7. Biochemical Assays

The measurement of ACh, 5-HT, DA, and NA contents were performed in strict accordance with the instructions of the ELISA kits. The measurement of the activities of T-SOD, CAT, and LPO, and the MDA content were performed in strict accordance with the instructions of the kits. The optical density of each sample had been detected by using a microplate reader.

### 2.8. Western Blot Analysis

After adding a protease inhibitor, brain tissues were prepared on ice. The supernatants were centrifuged at 4000 g, and the tests were carried out strictly according to the instructions of the kit. Total protein was extracted from brain tissues in each group, and protein was quantified according to the bicinchoninic acid protein quantification kit instructions (Nanjing Jiancheng, China). Proteins were separated by 10% SDS–PAGE, transferred by electrophoresis onto polyvinylidene fluoride membranes, incubated with TBST containing 5% nonfat milk at room temperature for 1 h, and then washed 5 times with TBST for 5 min each. Diluted Nrf2 (1 : 500), KEAP1 (1 : 1000), HO-1 (1 : 1000), and *β-*Actin antibodies (1 : 5000) were added separately, and the membranes were incubated overnight at 4°C. The next day, the membranes were rinsed 5 times with TBST for 5 min each, and the corresponding horseradish peroxidase-labelled secondary antibody (1 : 5000) was added. The membranes were incubated for 1 h at room temperature and then rinsed 5 times in TBST for 5 min each time. The films were rapidly developed according to the instructions of the electron chemiluminescence kit (New Cell & Molecular Biotech, China). ImageJ software was utilized for the quantitative analysis of images. Each experiment for each protein was repeated 3 times.

The article "Effect of Noni on Memory Impairment Induced by Hydrocortisone in Mice" was published in 2022. Journal: Evid Based Complement Alternat Med.

### 2.9. Statistical Analysis

Analysis was performed using SPSS (version 22.0, SPSS Inc., Chicago, IL, USA). The measurement data are presented as mean ± standard deviation ($\bar{x}$ ± *s*). One-way ANOVA followed by the Bonferroni method was adopted to compare the sample mean pairs. Values of *p* < 0.05 were considered statistically significant.

## 3. Results

### 3.1. Noni Had No Effect on Weight or the BI in Memory-Impaired Mice

During the experiment, the activity of the mice in each group was normal, and the hair colour was normal. There was no significant difference in body weight or the brain index after modelling and medication (*p* > 0.05). Hydrocortisone, noni, and ginseng had no effect on body weight or the brain index (Table 1).

### 3.2. Noni Ameliorated Ethological Behaviour in Memory-Impaired Mice

The step-down avoidance test and passive avoidance test results showed that both the incubation period and vanish period times in the control group were longer than those in the model group (*p* < 0.01). The error times and vanish error times in the control group were lower than those in the model group (*p* < 0.01). Compared with the model group, both the incubation period and the vanishing period times in the ginseng and high-dose groups were longer (*p* < 0.01). The error times and vanish error times in the ginseng and high-dose noni groups were lower (*p* < 0.01). Compared with the low-dose noni group, the incubation period and vanish period times in the high-dose noni group were longer (*p* < 0.01). The error times and vanish error times in the high-dose noni group were lower (*p* < 0.01) (Tables 2 and 3).

### 3.3. Pathology of the Brain Tissue of Mice in Each Group

In the control group, the neurons in the CA3 area of the hippocampus were arranged in a compact and orderly manner. Compared with the control group, the vertebral cells in the CA3 area of the hippocampus in the model group were loosely arranged, with obvious deep staining or pyknosis. Compared with the model group, the arrangement of neurons in the hippocampal CA3 area of each treatment group was slightly compact, and the deep staining and pyknosis of the cells were reduced (Figure 1).

The article "Effect of Noni on Memory Impairment Induced by Hydrocortisone in Mice" was published in 2022. Journal: Evid Based Complement Alternat Med.

The left side of each picture is 10*x* light mirror field of view, and the right side is 100*x* light mirror field of view.

### 3.4. Noni Altered Neurotransmitters in the Brains of Memory-Impaired Mice

Compared with the control group, ACh, 5-HT, DA, and NA in the model group were significantly decreased (*p* < 0.01). Compared with the model group, the four neurotransmitters of the ginseng group, h-dose noni group and middle-dose group were significantly regained (*p* < 0.01 or *p* < 0.05). Compared with levels in the low-dose noni group, ACh, 5-HT, DA, and NA in the brain were significantly increased in the high-dose noni group (*p* < 0.01) (Table 4).

### 3.5. Noni Improved the Antioxygen Ability in Memory-Impaired Mice

Compared with the control group, all the enzymes in the model group were significantly decreased (*p* < 0.01), and MDA in the brain was significantly increased (*p* < 0.01). Compared with the model group, the ginseng group and high-dose noni group had restored levels of all the enzymes and showed a decrease in the MDA content. Compared with the levels in the low-dose noni group, T-SOD, CAT, and LPO in the brain were significantly increased in the high-dose noni group (*p* < 0.01) (Table 5).

### 3.6. Protein Expression in the Brain Tissue of Mice

Compared with expression in the control group, Nrf2, KEAP1, and HO-1 protein expression in the brain was significantly decreased in the model group (*p* < 0.05 or *p* < 0.01). Compared with that in the model group, Nrf2, KEAP1, and HO-1 protein expression in the brain was significantly increased in the ginseng group and high-dose noni group (*p* < 0.05 and *p* < 0.01). Compared with the expression in the low-dose noni group, Nrf2, KEAP1, and HO-1 protein expression in the brain was significantly increased in the high-dose noni group (*p* < 0.01) (Figure 2).

## 4. Discussion

With the development of society, the problem of memory impairment is becoming increasingly serious and has gradually become a global problem. It is estimated that 150 million people will suffer from dementia by 2030. At present, there is no specific drug for memory impairment. As a kind of fruit with special functions, noni has the potential to become a product to improve memory. Hydrocortisone has been reported to cause memory impairment in rodents and to affect autobiographical memory recall in humans by accelerating impairment and ageing in the hippocampus, which loses large pyramidal neurons [17, 18]. Memory impairment caused by hydrocortisone is used as a drug tool to improve memory research. Thus, we used hydrocortisone to establish an animal model of memory impairment and observed the memory impairment ameliorating effects of noni to investigate its mechanism. Ginseng, as a traditional Chinese herbal drug, has been used to improve memory for hundreds of years. Modern research shows that ginseng can improve memory [19]. Thus, ginseng was selected as a positive control drug in our experience for comparison with noni. The selection of the dose of noni was based on our previous studies [20]. Our experience shows that after 14 days of modelling, there were significant differences between the control group and the model group, which showed changes in oxidative stress indices and behavioural changes. After the application of ginseng or noni, the overall levels of Nrf2, KEAP1, and HO-1 were significantly higher than those of the model group. In addition, Nrf2 was increased and the level of oxidative stress was reduced. Nrf2 activates the transcription and translation of phase II detoxification enzymes, such as SOD, CAT, and LPO. As a result, the expression of these enzymes in the brain tissue is increased, and neurotransmitters in the brain are also restored, which has a protective effect on neurons. Furthermore, memory impairment was recovered. The results of HE staining showed that the pyramidal cells of the hippocampal CA3 region in the model group were loosely arranged and had obvious hyperchromasia or pyknosis. The results indicated that there was an obvious neuron loss after hydrocortisone injection. After administration of ginseng or noni, the hyperchromasia and pyknosis of vertebral cells in the CA3 area of the hippocampus were alleviated, indicating that ginseng or noni could inhibit the loss of neurons in mice. The behaviour results of the step-down test and passive avoidance test showed that hydrocortisone induced severe memory impairment in mice. Ginseng or noni could improve the memory of mice.

The article "Effect of Noni on Memory Impairment Induced by Hydrocortisone in Mice" was published in 2022. Journal: Evid Based Complement Alternat Med.

Memory is an important function of the human brain, and its physiological function mainly depends on the hippocampal CA3 area [21]. The structural basis of memory is the limbic system, in which neurons in the hippocampal CA3 area are important cells involved in memory function [22]. Pyramidal cells are the main projection neurons in the hippocampus. The number of synapses in pyramidal cells is very large, which is the structural basis of information transmission between neurons [23]. Therefore, pyramidal cells in the hippocampal CA3 area are closely related to memory.

The step-down test and passive avoidance test are the most commonly used experimental methods to test learning and memory in mice. The step-down test uses the latency of staying on the platform and escaping to the platform, as well as the error times for jumping back to the click area as the index to investigate the learning and memory function of mice. The passive avoidance test is an inhibitory avoidance task designed based on the fact that mice tend to go towards the dark and avoid the light. It reflects the function of the hippocampus [24]. Some studies have shown that the decline in memory function in mice may be related to the decrease in the CAT and LPO contents in the brain [25].

Current studies have shown that Nrf2 is involved in different signalling pathways, including the Nrf2/HO-1 signalling pathway [26], KEAP1/Nrf2 signalling pathway [27], Nrf2/PINK1 mitochondrial signalling pathway [28], Nrf2/MAPK signalling pathway [29], and PI3K/Akt/Nrf2 signalling pathway [30]. Nrf2-involved signalling pathways regulate the antioxidant defence system and play an important role in antioxidant species under regulatory conditions, promoting defence and even resisting more damage. Nrf2 is expressed in various organs of the body and participates in the protection and defence processes of various systems of the body. The Nrf2/HO-1-signalling pathway is a potential target to prevent memory damage by regulating the redox balance of the brain. Oxidative stress is considered a sign of memory loss and a risk factor for memory impairment. Exogenous antioxidants can be supplemented to reduce the degree of oxidative stress. In particular, Nrf2 is an ideal choice to improve the endogenous antioxidant defence strategy pathway. It is a suitable choice for studying the molecular redox balance in cells, as it acts as a master antioxidant that regulates phase II detoxification. Under physiological conditions, Nrf2 binds to KEAP1 in the cytoplasm. When the level of endogenous or exogenous ROS increases, Nrf2 and KEAP1 dissociate, and phosphorylated Nrf2 is transferred to the nucleus, which combines with the small Maf protein in the nucleus to form a dimer, which starts the transcription of phase II detoxification enzymes, including HO-1, LPO, SOD, and CAT [31, 32]. After translation, the intracellular phase II detoxification enzymes increase, accelerating the scavenging and metabolism of ROS, and restoring the internal environment of cells. HO-1 plays an antioxidant role by removing oxygen-free radicals by generating carbon monoxide and free iron. It can eliminate the memory damage caused by hydrocortisone, inhibit lipid peroxidation of the cell membrane, and protect tissue cells from oxidative damage. According to previous research, deacetylasperulosidic acid and asperulosidic acid, kinds of iridoid, are the main active substances of noni [33, 34], which has antioxidant effects by increasing catalase activity in rats [35] and exists in *Ligustrum lucidum* Ait [36] and *Cornus officinalis* Sieb [37]. The noni fruit water extract 3and noni fruit polysaccharide alleviated oxidative stress and inflammation in mice under a high-fat diet [38]. Comparing to the current treatments of memory impairment such as memantine hydrochloride and donepezil, they had cardiac circulation system side effects [39]. Noni as a functional food can regulate Nrf2/KEAP1/HO-1 signalling pathway proteins and affect the synthesis of downstream oxidative stress proteins. Noni can reduce the oxidative stress damage of nerve cells and increase neurotransmitter levels in the brain, which ameliorates the memory impairment induced by hydrocortisone. Noni thus plays a protective role in mice.

The article "Effect of Noni on Memory Impairment Induced by Hydrocortisone in Mice" was published in 2022. Journal: Evid Based Complement Alternat Med.

## 5. Conclusion

Based on these findings, it can be suggested that noni might be a powerful antioxidant and protect nerve cells. Noni may possess a potential benefit for the treatment of memory impairment [40].

## Figures and Tables

**Figure 1:** Mice brain tissue of HE staining (×10, ×100).

**Figure 2:** Nrf2, KEAP1, and HO-1 protein expression in brain tissue of mice in each group ($\bar{x}$ ± *s*, *n* = 3). Notes: vs. control group *p*_ _^*∗*^ < 0.05; vs. model group *p*_ _^#^ < 0.05.

**Table 1:** Weight of mice and BI ($\bar{x}$ ± *s*, *n* = 8).

Group	7d weight (g)	14d weight (g)	BI (%)
Control	25.6 ± 0.9	42.4 ± 2.1	0.7 ± 0.1
Model	25.6 ± 0.6	39.5 ± 2.2	0.8 ± 0.1
Ginseng	25.3 ± 0.9	39.0 ± 4.2	0.8 ± 0.1
H-Noni	25.3 ± 0.6	38.5 ± 3.5	0.8 ± 0.0
M-Noni	25.6 ± 1.1	39.0 ± 2.7	0.8 ± 0.1
L-Noni	25.1 ± 0.9	38.1 ± 3.1	0.8 ± 0.0

**Table 2:** Effects of noni on the step-down avoidance test in mice ($\bar{x}$ ± *s*, *n* = 8).

Group	Incubation period (s)	Error time	Vanish period (s)	Vanish error time
Control	145.9 ± 2.9	3.0 ± 2.1	181.8 ± 4.7	1.5 ± 0.9
Model	72.1 ± 8.2 ^*∗*^ ^*∗*^	5.9 ± 1.4 ^*∗*^ ^*∗*^	97.6 ± 6.0 ^*∗*^ ^*∗*^	4.1 ± 1.1 ^*∗*^ ^*∗*^
Ginseng	99.3 ± 12.9^##^	2.5 ± 1.3^##^	155.6 ± 8.4^##^	1.6 ± 0.7^##^
H-Noni	120.4 ± 11.0^##△△^	3.0 ± 0.9^##△△^	163.4 ± 9.2^##△△^	1.5 ± 0.9^##△△^
M-Noni	90.1 ± 11.3^##△△^	3.1 ± 1.7^##△△^	135.3 ± 7.4^##△△^	3.0 ± 0.8^#^
L-Noni	79.3 ± 6.2	4.6 ± 1.5	104.1 ± 10.6	4.0 ± 0.8

Notes: vs. control group *p*_ _^*∗∗*^ < 0.01; vs. model group *p*_ _^#^ < 0.05, *p*_ _^##^ < 0.01; vs. L-noni group *p*_ _^ΔΔ^ < 0.01.

The article "Effect of Noni on Memory Impairment Induced by Hydrocortisone in Mice" was published in 2022. Journal: Evid Based Complement Alternat Med.

**Table 3:** Effects of noni on the passive avoidance test in mice ($\bar{x}$ ± *s*, *n* = 8).

Group	Incubation period (s)	Error time	Vanish period (s)	Vanish error time
Control	49.5 ± 6.5	2.0 ± 1.7	132.3 ± 8.3	2.0 ± 1.7
Model	31.5 ± 6.1 ^*∗*^ ^*∗*^	4.1 ± 1.1 ^*∗*^ ^*∗*^	80.3 ± 6.2 ^*∗*^ ^*∗*^	4.0 ± 1.2 ^*∗*^ ^*∗*^
Ginseng	58.1 ± 6.4^##^	1.9 ± 0.8^##^	115.8 ± 10.4^##^	2.1 ± 1.0^##^
H-noni	46.4 ± 6.7^##△△^	2.0 ± 1.1^##△△^	124.9 ± 14.2^##△△^	2.4 ± 1.2^##△△^
M-noni	38.5 ± 5.0^#△△^	3.9 ± 0.8	123.0 ± 5.1^##△△^	3.6 ± 0.7
L-noni	29.0 ± 4.4	4.4 ± 0.7	108.0 ± 9.0^##^	4.1 ± 1.0

Notes: vs. control group *p*_ _^*∗∗*^ < 0.01; vs. model group *p*_ _^##^ < 0.01; vs. L-noni group *p*_ _^ΔΔ^ < 0.01.

**Table 4:** Expression of neurotransmitters in brain ($\bar{x}$ ± *s*, *n* = 8).

Group	ACh (pmol/g)	5-HT (ng/g)	DA (ng/g)	NA (ng/g)
Control	11.34 ± 0.86	7.04 ± 0.45	25.85 ± 2.96	37.68 ± 8.11
Model	7.65 ± 0.93 ^*∗*^ ^*∗*^	4.97 ± 0.24 ^*∗*^ ^*∗*^	16.10 ± 1.18 ^*∗*^ ^*∗*^	27.39 ± 1.84 ^*∗*^ ^*∗*^
Ginseng	13.86 ± 2.23^##^	6.61 ± 0.55^##^	26.72 ± 5.28^##^	36.40 ± 5.50^##^
H-noni	13.79 ± 2.87^##△△^	6.66 ± 0.71^##△△^	26.40 ± 2.59^##△△^	41.00 ± 6.91^##△△^
M-noni	10.57 ± 1.68^##^	5.74 ± 0.43^*∗∗*##^	21.06 ± 4.69^#^	35.46 ± 3.90^#^
L-noni	9.39 ± 1.31	5.52 ± 0.32 ^*∗*^ ^*∗*^	19.18 ± 3.51	30.26 ± 1.38

Notes: vs. control group *p*_ _^*∗∗*^ < 0.01; vs. model group *p*_ _^#^ < 0.05, *p*_ _^##^ < 0.01; vs. L-noni group *p*_ _^ΔΔ^ < 0.01.

**Table 5:** Expression of T-SOD, CAT, LPO, and MDA in the brain ($\bar{x}$ ± *s*, *n* = 8).

Group	T-SOD (U/mgprot)	CAT (U/mgprot)	LPO (U/mgprot)	MDA (mgprot/ml)
Control	141.37 ± 13.07	3.94 ± 0.25	0.57 ± 0.13	2.08 ± 0.40
Model	104.96 ± 10.01 ^*∗*^ ^*∗*^	3.29 ± 0.23 ^*∗*^ ^*∗*^	0.27 ± 0.06 ^*∗*^ ^*∗*^	2.58 ± 0.20 ^*∗*^ ^*∗*^
Ginseng	139.41 ± 20.76^##^	3.70 ± 0.42	0.54 ± 0.09^##^	2.21 ± 0.42^#^
H-noni	141.69 ± 18.19^##△△^	4.99 ± 0.66^##△△^	0.56 ± 0.11^##△△^	1.81 ± 0.38^##^
M-noni	111.23 ± 11.71	3.71 ± 0.55	0.35 ± 0.12	1.89 ± 0.23^##^
L-noni	110.35 ± 14.14	3.58 ± 0.34	0.32 ± 0.06	2.07 ± 0.23^##^

Notes: vs. control group *p*_ _^*∗∗*^ < 0.01; vs. model group *p*_ _^#^ < 0.05, *p*_ _^##^ < 0.01; vs. L-noni group *p*_ _^ΔΔ^ < 0.01.

## Data Availability

The datasets generated and/or analysed during the current study are available in the [Zhang, Rui (2022): Noni database. figshare. Dataset.] repository [https://doi.org/10.6084/m9.figshare.20019782.v1].
